# Applications of bioconvection for tiny particles due to two concentric cylinders when role of Lorentz force is significant

**DOI:** 10.1371/journal.pone.0265026

**Published:** 2022-05-03

**Authors:** Lei Zhang, V. Puneeth, Muhammad Ijaz Khan, Essam Roshdy El-Zahar, N. Manjunath, Nehad Ali Shah, Jae Dong Chung, Sami Ullah Khan, M. Imran Khan

**Affiliations:** 1 Yellow River Institute of Hydraulic Research, YRCC, Zhengzhou, China; 2 Henan Engineering Research Center of Hydropower Engineering Abrasion Test and Protection, Zhengzhou, China; 3 Department of Mathematics, CHRIST (Deemed to be University), Bengaluru, India; 4 Department of Mathematics and Statistics, Riphah International University, Islamabad, Pakistan; 5 Department of Mathematics, College of Science and Humanities in Al-Kharj, Prince Sattam Bin Abdulaziz University, Al-Kharj, Saudi Arabia; 6 Department of Basic Engineering Science, Faculty of Engineering, Menoufia University, Shebin El-Kom, Egypt; 7 Department of Sciences and Humanities, CHRIST (Deemed to be University), Bengaluru, India; 8 Department of Mechanical Engineering, Sejong University, Seoul, Korea; 9 Department of Mathematics, COMSATS University Islamabad, Sahiwal, Pakistan; 10 Division of Sustainable Development, College of Science and Engineering, Hamad Bin Khalifa University, Qatar Foundation, Doha, Qatar; Stellenbosch University, SOUTH AFRICA

## Abstract

The bioconvection flow of tiny fluid conveying the nanoparticles has been investigated between two concentric cylinders. The contribution of Lorenz force is also focused to inspect the bioconvection thermal transport of tiny particles. The tiny particles are assumed to flow between two concentric cylinders of different radii. The first cylinder remains at rest while flow is induced due to second cylinder which rotates with uniform velocity. Furthermore, the movement of tiny particles follows the principle of thermophoresis and Brownian motion as a part of thermal and mass gradient. Similarly, the gyro-tactic microorganisms swim in the nanofluid as a response to the density gradient and constitute bio-convection. The problem is modeled by using the certain laws. The numerical outcomes are computed by using RKF -45 method. The graphical simulations are performed for flow parameters with specific range like 1≤Re≤5, 1≤*Ha*≤5, 0.5≤*Nt*≤2.5, 1≤*Nb*≤3, 0.2≤*Sc*≤1.8, 0.2≤*Pe*≤1.0 and 0.2≤Ω≤1.0. It is observed that the flow velocity decreases with the increase in the Hartmann number that signifies the magnetic field. This outcome indicates that the flow velocity can be controlled externally through the magnetic field. Also, the increase in the Schmidt numbers increases the nanoparticle concentration and the motile density.

## 1. Introduction

A nanofluid is a novel class of fluids in which metallic or nonmetallic nanoparticles are scattered over the base fluid. These nanofluids are known for their special heat transfer properties like the presence of nanoparticles pronounced the reflective thermal aspect of base materials [1]. This special property makes these fluids applicable for several engineering applications such as coolants in automobiles, nuclear reactors, solar heaters etc. Some of the special properties of nanoparticles are high specific surface area, higher dispersion stability, reduced particle clogging, and many adjustable properties including thermal conductivity and surface wettability [2]. In this regard, Sheikholeslami [3] studied the impact of porosity and Lorentz force on the heat transfer of nanofluid using Darcy law. Bhamani et al. [4] made contributions for growing heating aspect for turbulent flow of nanofluid inside a pipe. Alrashed et al. [5] modelled a system that describes the flow and the thermal performance of nanofluid comprising of water and MWCNT. Abbas et al. [6] scrutinized the entropy generation in the fully developed flow of nanofluid subjected to velocity slip. Nadeem et al. [7] analyzed the heat transfer characteristics of hybrid nanofluid flowing over a curved surface. The nanomaterials various improved migrated phenomenon with subclass of base fluids was directed in communications Puneeth et al. [8, 9]. These continuations on the analysis of heat transfer of single-phase and double phase nanofluid were extended to ternary nanofluid by Manjunatha et al. [10] which comprises of a base fluid and three different classes of nanoparticles. Song et al. [11] reported the thermal distribution of alumina and copper nanomaterials with ethylene glycol and water base fluid. Oke et al. [12] expressed the role of Coriolis force to express the thermal experience of alumina nanoparticles with diameter 47nm. Animasaun et al. [13] presented the thermo-haphazard prospective of nanoparticles with diverse thermal properties. The inclusion of tiny nanoparticles in different kind of base liquids with meta investigations was directed by Wakif et al. [14].

Pattern-forming convection movements established in suspensions of paddling microorganisms is known as bio-convection. In liquid suspensions of floating microorganisms, the cellular streaming trend was found wherein fluid flow motions proceed downwards in places where elevated levels of microorganisms develop and swim upwards in regions of low concentration. This sort of pattern is determined by factors including the depth of the suspension, as well as the quantity and mobility of the organisms. Khan et al. [15] used the Cattaneo-Christov model to analyze the double diffusion in the nanofluid flow containing motile cells. This was further followed by Yahya et al. [16] to explore the bio-convection in Williamson nanofluid. Similarly, Puneeth et al. [17] considered the bio-convective flow of Williamson nanofluid past a Riga plate. Shi et al. [18] analyzed the impact of activation energy and gyro-tactic microorganisms in enhancing the thermal performance of magneto-cross nanofluid. Waqas et al. [19] performed simulations using numerical methods to analyze the impact of microorganisms swimming in a non-Newtonian nanofluid subject to the magnetic field. Further, Koriko et al. [20] analyzed the process of bio-convection comprising the implosion of microorganisms in a thixotropic nanofluid. Puneeth et al. [21] discussed the homogeneous and heterogeneous chemical reactions with the quartic autocatalysis for the flow of micropolar nanofluid flowing in a channel subjected to thermal radiation for microorganism interference. Azam et al. [22] evaluated the impact of nonlinear radiation in the flow of nanofluid under the influence of motile cells. Balla et al. [23] encountered the chemical reaction aspect while reporting the bioconvection phenomenon for oxytactic microorganisms. Makinde and Animasaun [24] performed the determination of bioconvection pattern subject to autocatalysis reactive species in the upper regime of paraboloid. The fluctuation in bioconvective properties of nanofluids with influence of nonlinear radiative phenomenon in paraboloid revolution was visualized in the work of Makinde and Animasaun [25]. Khan et al. [26] rolled out the impact of Navier slip for nanofluids flow with microorganisms. Khan and Makinde [27] conveyed the heat transfer improvement for nanofluids flow with bioconvection enrolment.

The motion of suspended matter across a fluid in the presence of a temperature gradient is known as thermophoresis. A study to interpret the role of thermophoresis on particle migration and concentration distribution discovered that the concentration distribution gets more non-uniform as the particle size increases. Meanwhile, thermophoresis accentuates non-uniformity in the concentration distribution, with a stronger effect at higher mean concentrations [28]. Many researchers have explored the flow with thermophoresis and Brownian motion as they play an important role in the analysis of heat and mass transfer. For instance, Sheikholeslami et al. [29] studied the impact of magnetic force for tiny particles imposed two cylinders having circular orientation. Mirzaeyan and Toghraie [30] investigated the laminar flow of nanofluid between porous cylinders. Arif et al. [31] justified importance of *GO* nanoparticle in the *MoS*_2_−*H*_2_*O* nanofluid for enhancing its thermal performance. Abbas et al. [32] analyzed the impact of magnetic field on the velocity of nanofluid flowing past a non-linear stretching sheet. Reddy et al. [33] employed the Cattaneo-Christov heat flux model to examine the thermal characteristics of nanofluid flowing past a swirling cylinder. Biswal et al. [34] deterimned numerical simulation to investigate the flow of a nanofluid in a semi-porous channel subjected to the magnetic field. Khan et al. [35] discussed the impact of Joule heating referring to interaction of nano-compounds past a swirling cylinder under the influence of Lorentz force. Aghamiri et al. [36] designed a mathematical model that describes the impact of forced convection on the flow of Ferro-nanofluid flowing in a microchannel consisting of rotating cylinders. Bouzerzour et al. [37] discussed natural convection in a nanofluid flowing in an annular space formed due to the separation between confocal elliptic cylinders at different geometric positions. Ch et al. [38] claimed thermophoresis inspection of Walter’s B nanofluid subject to interaction of buoyancy forces. Khan and Ali [39] worked out the thermophoresis model based on nanofluid properties by using Eyring-Powell fluid model. The thermal statement and role of thixotropic nanomaterials incorporating the thermo-diffusion phenomenon for Riga configuration was addressed by Khan et al. [40].

After presenting a comprehensive literature survey, it has been noticed that bioconvection aspect of nanofluid with various flow configurations have been available. However, the bioconvection applications of tiny fluid conveying the nanoparticles between two concentric cylinders different radii is not focused yet. Moreover, the contribution of Lorentz force for bio-convective model is another important task which is addressed in this model. The flow though moving cylinder is interesting topic and some continuations are performed by researchers [41–50]. This investigation presents the answer of following thermal flow questions:

- Which mathematical model is used to inspect the bioconvection of tiny particles moving between concentric cylinders having different radii?
- How heat and mass transfer process fluctuated with interaction of tiny fluid conveying the nanoparticles?
- What is contribution of Lorentz force to improve the heating phenomenon?
- How thermophoresis and Brownian motion parameters pays role to enhance the thermal process?

## 2. Mathematical model

A laminar flow of a Newtonian fluid containing the nanoparticles in the presence of gyro-tactic microorganisms is assumed to flow between two concentric cylinders. Each of these cylinders are of radii *R*_1_ and *R*_2_ such that *R*_1_>*R*_2_. The cylinder with radius *R*_2_ is assumed to be stationary and is enclosed in the cylinder of radius *R*_1_, whose angular momentum is *ω*_1_. The presence of microorganisms in the system stabilizes the dilute nanoparticle suspension and prevent sedimentation in the system. The dilute nanoparticle suspension is assumed which no fluctuation of movement of microorganisms within the system. This enables the microorganisms to move easily and constitute the macroscopic phenomena termed bio-convection. Thermophoresis and Brownian motion prospective of tiny particles is examined in view of Buongiorno thermal model. Hence, these two slip mechanisms are included in the mathematical model so that the results that are obtained will be close to practicality. Furthermore, the cylinders of radii *r*_1_ and *r*_2_ are maintained at a temperature *T*_1_ and *T*_2_ respectively along with the concentration *C*_1_ and *C*_2_ and the motile density *N*_1_ and *N*_2_ respectively. The flow configuration is shown in Fig 1 using cylindrical coordinates.

**Fig 1:** Schematic flow diagram.

The exploration of thermal model for all constraints is presented via following equations [36, 37, 46]:

$$\bar{u}\frac{d\bar{u}}{d\bar{r}}=\nu [\frac{d^{2}\bar{u}}{d{\bar{r}}^{2}}-\frac{\bar{u}}{{\bar{r}}^{2}}+\frac{1}{\bar{r}}\frac{d\bar{u}}{d\bar{r}}]-\frac{\sigma B_{0}^{2}}{\rho }\bar{u},$$ (1)

$$\bar{u}\frac{dT}{d\bar{r}}=\alpha [\frac{d^{2}T}{d{\bar{r}}^{2}}+\frac{1}{\bar{r}}\frac{dT}{d\bar{r}}]+\frac{{\left(\rho C_{p}\right)}_{f}}{\left(\rho C_{p}\right)}[D_{B}\frac{dT}{d\bar{r}}\frac{dC}{d\bar{r}}+\frac{D_{T}}{T_{2}}{\left(\frac{dT}{d\bar{r}}\right)}^{2}],$$ (2)

$$\bar{u}\frac{dC}{d\bar{r}}=D_{B}[\frac{d^{2}C}{d{\bar{r}}^{2}}+\frac{1}{\bar{r}}\frac{dC}{d\bar{r}}]+\frac{D_{T}}{T_{2}}[\frac{d^{2}T}{d{\bar{r}}^{2}}\frac{1}{\bar{r}}\frac{dT}{d\bar{r}}],$$ (3)

$$\bar{u}\frac{dN}{d\bar{r}}=D_{N}[\frac{d^{2}N}{d{\bar{r}}^{2}}+\frac{1}{\bar{r}}\frac{dN}{d\bar{r}}]-\frac{bW_{c}}{C_{1}-C_{2}}\frac{d}{d\bar{r}}[N\frac{dC}{d\bar{r}}],$$ (4)

with

$$\begin{array}{c} \bar{u}=\omega_{1}r_{1},\;T=T_{1},\;C=C_{1},\;N=N_{1},\;\mathrm{at}\;\bar{r}=r_{1},\;\\ \bar{u}=0,\;T=T_{2},\;C=C_{2},\;N=N_{2},\;\mathrm{at}\;\bar{r}=r_{2}, \end{array}\}$$ (5)

The non-dimensionless form of model is [36, 37, 46]:

d2udr2+1rdudr−Reududr−((Ha)2(1−ε)2+1r2)u=0, (6)

d2θdr2+1rdθdr−RePrudθdr+Nbdϕdrdθdr+Nt(dθdr)2=0, (7)

d2ϕdr2+1rdϕdr−ReScudϕdr+NtNb(d2θdr2+1rdθdr)=0, (8)

d2Xdr2+1rdXdr−ReSbudXdr−Pe(dXdrdCdr+Xdϕdr+Ωd2ϕdr2)=0, (9)

The corresponding boundary conditions are

$$\begin{array}{c} u=1,\;\theta =1\;\phi =1\;X=1\;r=\varepsilon ,\;\\ u=0,\;\theta =0\;\phi =0\;X=0\;r=1. \end{array}\}$$ (10)

The dimensionless parameters involved in this study are defined as

$$\begin{array}{c} \varepsilon =\frac{r_{1}}{r_{2}},\;r=\frac{\bar{r}}{r_{2}},\;Ha=B_{0}(r_{2}-r_{1})\frac{\sigma B_{0}^{2}}{\rho },\;\theta =\frac{T-T_{1}}{T_{0}-T_{1}},\;\phi =\frac{C-C_{1}}{C_{0}-C_{1}},\;X=\frac{N-N_{1}}{N_{0}-N_{1}},\;\\ Re=\frac{\Omega r_{1}r_{2}}{\nu },\;\mathrm{Pr}=\frac{\nu }{\alpha },\;Nt=\frac{\tau D_{T}(T_{0}-T_{1})}{\alpha T_{1}},\;Nb=\frac{\tau D_{B}(C_{0}-C_{1})}{\alpha },\;\\ Sc=\frac{\nu }{D_{B}},\;Sb=\frac{\nu }{D_{N}},\;Pe=\frac{bW_{c}}{D_{N}},\;\Omega =\frac{N_{2}}{N_{1}-N_{2}},\;u=\frac{\bar{u}}{\omega_{1}r_{1}}. \end{array}\}$$ (11)

## 3. Solution methodology

The transformed Eqs (6)–(9) along with the boundary conditions (10) are remodeled to initial value problem (IVP). This is further simulated with interpretation of well-known RKF -45 method in acquaintance with the shooting method. For the computation purpose, the infinite boundary conditions are considered at *η* = 10 and the accuracy of the solution is set to the order of 10^−5^. The proper step size is determined in this method for ensuring the validity. Further, these two approximations are compared and if they hold a close agreement with each other than the approximation is considered valid. The whole process is repeated if the approximations obtained do not match each other and the computation is repeated till the desired accuracy is obtained.

## 4. Results and discussion

RKF -45 is used to examine the flow of nanofluid between two concentric cylinders in the presence of self-propelled microorganisms. Using appropriate relationships, the equations are non-dimensionalised. The solution was achieved using RKF -45. The outcomes of this study are interpreted through graphs ((2a)-(5d)) and Tables 1 and 2.

**Table 1:** Variations of quantities of physical interest for the changes in Re and *Ha*.

Parameter	Range	$-{\left(\frac{du}{dr}\right)}_{r=0}$	$-{\left(\frac{d\theta }{dr}\right)}_{r=0}$	$-{\left(\frac{d\phi }{dr}\right)}_{r=0}$	$-{\left(\frac{dX}{dr}\right)}_{r=0}$
Re	1	6.019791941	0.114981271	2.455937464	3.294764449
	2	5.599051794	0.033347737	1.570841211	1.789029468
	3	5.188232292	0.008195391	0.928568857	0.800785493
	4	4.789171985	0.001681899	0.503667618	0.252470081
	5	4.404083642	0.000282309	0.248382388	0.013075776
Ha	1	5.260641448	0.098887375	2.350184677	3.120977258
	2	6.019791941	0.114981271	2.455937464	3.294764449
	3	7.010034918	0.134403776	2.572311573	3.487258489
	4	8.098824067	0.153031691	2.675925633	3.660256028
	5	9.234128219	0.169444086	2.762766988	3.806829769

**Table 2:** Variations of quantities of physical interest for the changes in *Sc*, *Nb* and *Nt*.

Parameter	Range	$-{\left(\frac{d\theta }{dr}\right)}_{r=0}$	$-{\left(\frac{d\phi }{dr}\right)}_{r=0}$	$-{\left(\frac{dX}{dr}\right)}_{r=0}$
Sc	1	0.106610988	3.185041421	3.742403689
	2	0.110749611	2.801801917	3.507260711
	3	0.114981271	2.455937464	3.294764449
	4	0.119287931	2.145470405	3.103745486
	5	0.123651544	1.868213341	2.932904232
Nb	1	0.482348184	3.112881171	3.700386708
	2	0.241850059	2.630081554	3.402457446
	3	0.114981271	2.455937464	3.294764449
	4	0.052410192	2.364185944	3.237914973
	5	0.023120414	2.307734571	3.202886897
Nt	0.5	0.114981271	2.455937464	3.294764449
	1.0	0.077230578	2.824710126	3.522508617
	1.5	0.051498855	3.191753058	3.748817773
	2.0	0.034117987	3.555669601	3.972797117
	2.5	0.022471965	3.916123096	4.194239191

Fig 2(A)–2(D) shows the impact of Reynolds number (Re) on the nanofluid flow profiles. Following the physical dynamic of Reynolds number, inertial forces grow up when Reynolds number is higher. Such forces show their major impact at the boundary region. As the value of Re goes higher, the viscous force becomes less significant, and the fluid will thus be less viscous and result in faster flow. The up-raise change in velocity due to Re is noted in Fig 2(A) Moreover, the temperature rate of tiny particles increases due to the friction created within the fluid due to its faster flowing rate as shown in Fig 2(B). Similarly, the Fig 2(C) and 2(D) indicated that improvement assigning to Reynolds number enhances the mass concentration and the motile density respectively.

**Fig 2:** The impact of Reynolds number on the fluid profiles.

The Hartmann number (*Ha*) is the ratio of electromagnetic forces to the viscous forces which measures the significance of drag forces resulting from electromagnetic induction and viscous forces. The impact of this parameter is shown in Fig 3(A)–3(D). The velocity of the nanofluid flow is seen to be reduced in Fig 3(A) because of the strong Lorentz force produced. This force acts against the flow and opposes the motion of the fluid by creating friction. Also, the friction thus created will generate additional heat within the nanofluid as a result more impressive temperature field is noted (Fig 3(B)) for higher values of *Ha*. Due to the slow movement of nanofluid, the nanoparticles and microorganisms accumulate at the boundary layer. The improved change in concentration and microorganism profile is noticed in Fig 3(C) and 3(D).

**Fig 3:** The impact of Hartmann number on the fluid profiles.

The impact of thermophoresis (*Nt*) on *θ*(*r*) and *ϕ*(*r*) is shown in Fig 4(A) and 4(B) respectively. The increase in the *Nt* parameter causes the nanoparticles to move from a hotter region to a colder and the nanoparticles dissipate heat into the fluid. As a consequence, the temperature of the nanofluid increases as shown in Fig 4(A). Meanwhile, the movement of nanoparticles becomes faster with the increase in Nt as a result, *ϕ*(*r*) at the boundary layer gowsup as reflected in Fig 4(B). Further, the temperature of the nanofluid increases due to the heat generated because of the collision of nanoparticles. Thus increment with increasing trend in referred to Fig 4(C) the zigzag motion of nanoparticles increases with the increase in Nb. During this zigzag motion, the nanoparticles colloid each other and move away from the boundary region as a result the nanoparticle concentration decreases as depicted in Fig 4(D).

**Fig 4:** The impact of Nt and Nb on the thermal and concentration profiles.

The impact of the Schmidt numbers on the Φ(*r*) and *X*(*r*) is depicted in Fig 5(A) and 5(B) respectively. The Schmidt numbers are inversely proportional to the diffusivities of their corresponding profiles. As a result, as the concentration Schmidt number (*Sc*) increases, the diffusivity of the nanoparticles reduces, and Φ(*r*) at the boundary layer falls, as illustrated in Fig 5(A). As Sb increases, the motile density diffusivity falls, and the motile density at the border layer drops, as seen in Fig 5(B). Furthermore, as illustrated in Fig 5(C), increasing the Peclet number increases motile density at the border layer. When Ω upgrade, the microorganism profile declined as shown in Fig 5(D).

**Fig 5:** The impact of *Sc*, *Pe* and Ω *on* Φ(*r*) and X(*r*).

The variations of wall shear surface force, local Nusselt number, Sherwood number and motile density number is tabulated in Tables 1 and 2 for changes in the fluid parameters. Table 1 displays the impact of Reynolds number and Hartmann number whereas, Table 2 shows the impact of Schmidt number and slip mechanisms. The increase in the Reynolds number resulted in a decrease in *Cf*_*r*_ *Nu*_*r*_, *Sh*_*r*_ and *Nn*_*r*_ and the same is tabulated in the first row of Table 1. Whereas, it was noticed that the higher values of *Ha* increased *Cf*_*r*_, *Nu*_*r*_, *Sh*_*r*_ and *Nn*_*r*_. Meanwhile, the increase in the Schmidt number increased the Nusselt number whereas it decreased the Sherwood number and motile density number. Furthermore, the increase in the values of *Nb*, decreased the values of *Nu*_*r*_, *Sh*_*r*_ and *Nn*_*r*_, but the higher values of *Nt* decreased the Nusselt number and enhanced Sherwood number and motile density number.

## 5. Conclusions

The applications of Lorentz force for bioconvection transport of tiny fluid conveying tiny particles due to two concentric cylinders is presented. For nanofluid flow, the concentric cylinders attained same center but different radius. The governing equations are made dimensionless using appropriate relationships for which simulations have been performed via RKF-45 method. Some of the major outcomes of the study are:

➢ The increment in Reynolds number enhanced the nanoparticle concentration and motile density profiles.
➢ The Hartmann number is dominant over the fluid flow and the higher values of *Ha* reduce the fluid flow.
➢ The enhanced flow velocity and heating phenomenon is noted for increasing the Reynolds number.
➢ The increase in the thermophoresis parameter enhances the thermal and mass profiles of the nanofluid.
➢ The greater values of Schmidt numbers enhance their corresponding profiles whereas the motile density decreases for higher Peclet numbers.

## Abbreviations

α: Thermal diffusivity
ν: Viscosity
Ω: Microorganisms difference number
ρ: Density
σ: Electrical conductivity
Pr: Prandtl number
b: Chemotaxis constant
Re: Reynolds number
Sb: Bio-convection Schmidt number
Sc: Schmidt number
*T*_1_, *T*_2_: Surface temperature
u: Velocity component
*W*_*c*_: Maximum cell swimming speed
Ha: Hartmann number
*N*_1_, *N*_2_: Motile density at the surface
Nb: Brownian motion parameter
Nt: Thermophoresis parameter
Pe: Peclet number
*ω*_1_: Angular momentum
*r*_1_, *r*_2_: radii
*B*_0_: Magnetic field strength
*C*_1_, *C*_2_: Nanoparticle concentration at the surface
*D*_*B*_: Brownian motion diffusivity
*D*_*N*_: Motile diffusivity
*D*_*T*_: Thermophoresis diffusivity

## References

[1] BhanvaseB. A., BaraiD. P., SonawaneS. S., ShirishH. and SonawaneN. K., Handbook of Nanomaterials for Industrial Applications. Elsevier, 2018, ch. 40, pp. 739–750.

[2] OkonkwoE. C., OshoI. W., AlmanassraI. W., AbdullatifY. M., and AnsariT. A., An updated review of nanofluids in various heat transfer devices, Journal of Thermal Analysis and Calorimetry, vol. 145, pp. 2817–2872, 2021.

[3] SheikholeslamiM., Application of darcy law for nanofluid flow in a porous cavity under the impact of lorentz forces, Journal of Molecular Liquids, vol. 266, pp. 495–503, 2018.

[4] BahmaniM. H., SheikhzadehG., ZarringhalamM., AkbariO. A., AlrashedA. A., ShabaniG. A. S., et al, Investigation of turbulent heat transfer and nanofluid flow in a double pipe heat exchanger, Advanced Powder Technology, vol. 29, no. 2, pp. 273–282, 2018.

[5] AlrashedA. A., AkbariO. A., HeydariA., ToghraieD., ZarringhalamM., ShabaniG. A. S., et al, The numerical modeling of water/fmwcnt nanofluid flow and heat transfer in a backwardfacing contracting channel, Physica B: Condensed Matter, vol. 537, pp. 176–183, 2018.

[6] AbbasS. Z., KhanM. I., KadryS., KhanW. A., Israr-Ur-RehmanM., and WaqasM., Fully developed entropy optimized second order velocity slip mhd nanofluid flow with activation energy, Computer Methods and Programs in Biomedicine, vol. 190, p. 105362, 2020. doi: 10.1016/j.cmpb.2020.105362 32032806

[7] NadeemS., AbbasN., and MalikM., Inspection of hybrid based nanofluid flow over a curved surface,Computer Methods and Programs in Biomedicine, vol. 189, p. 105193, 2020.10.1016/j.cmpb.2019.10519331981759

[8] PuneethV., ManjunathaS., MadhukeshJ., and RameshG., Three dimensional mixed convection flow of hybrid casson nanofluid past a non-linear stretching surface: A modified buongiorno’s model aspects, Chaos, Solitons & Fractals, vol. 152, p. 111428, 2021.

[9] PuneethV., ManjunathaS., MakindeO., and GireeshaB., Bioconvection of a radiating hybrid nanofluid past a thin needle in the presence of heterogeneous—homogeneous chemical reaction, Journal of Heat Transfer, vol. 143, no. 4, p. 042502, 2021.

[10] ManjunathaS., PuneethV., AnandikaR., and GireeshaB., Analysis of multilayer convective flow of a hybrid nanofluid in porous medium sandwiched between the layers of nanofluid, Heat Transfer, 2021.

[11] Ying-QingSongB.D.Obideyi, NehadAli Shah, AnimasaunI.L., MahrousY.M., JaeDongChung, Significance of haphazard motion and thermal migration of alumina and copper nanoparticles across the dynamics of water and ethylene glycol on a convectively heated surface, Case Studies in Thermal Engineering, Volume 26, August 2021, 101050.

[12] OkeA.S., AnimasaunI.L., MutukuW.N., KimathiM., Nehad Ali ShahS.Saleem, Significance of Coriolis force, volume fraction, and heat source/sink on the dynamics of water conveying 47 nm alumina nanoparticles over a uniform surface, Chinese Journal of Physics, Volume 71, June 2021, Pages 716–727.

[13] AnimasaunI.L., IbraheemR.O., MahantheshB., H.A.Babatunde A meta-analysis on the effects of haphazard motion of tiny/nano-sized particles on the dynamics and other physical properties of some fluids, Chinese Journal of Physics, Volume 60, August 2019, Pages 676–687

[14] WakifA., AnimasaunI.L., Satya NarayanaP.V., SarojammaG., Meta-analysis on thermo-migration of tiny/nano-sized particles in the motion of various fluids, Chinese Journal of Physics, Volume 68, December 2020, Pages 293–307

[15] KhanS. A., WaqasH., NaqviS. M. R. S., AlghamdiM., and Al-MdallalQ., Cattaneo-christov double diffusions theories with bio-convection in nanofluid flow to enhance the efficiency of nanoparticles diffusion, Case Studies in Thermal Engineering, vol. 26, p. 101017, 2021.

[16] YahyaA. U., SalamatN., HabibD., AliB., HussainS., and AbdalS., Implication of bio-convection and cattaneo-christov heat flux on williamson sutterby nanofluid transportation caused by a stretching surface with convective boundary, Chinese Journal of Physics, vol. 73, pp. 706–718, 2021.

[17] PuneethV., ManjunathaS., and GireeshaB., Bioconvection in buoyancy induced flow of williamson nanofluid over a riga plate-dtm-padé approach, Journal of Nanofluids, vol. 9, no. 4, pp. 269–281, 2020.

[18] ShiQ.-H., HamidA., KhanM. I., KumarR. N., GowdaR., PrasannakumaraB., et al, Numerical study of bio-convection flow of magneto-cross nanofluid containing gyrotactic microorganisms with activation energy, Scientific Reports, vol. 11, no. 1, pp. 1–15, 2021. doi: 10.1038/s41598-020-79139-8 34362971PMC8346499

[19] WaqasH., KhanS. A., AlghamdiM., AlqarniM., and MuhammadT., Numerical simulation for bioconvection flow of magnetized non-newtonian nanofluid due to stretching cylinder/plate with swimming motile microorganisms, The European Physical Journal Special Topics, pp. 1–18, 2021.

[20] KorikoO. K., ShahN. A., SaleemS., ChungJ. D., OmowayeA. J., and OreyeniT., Exploration of bioconvection flow of MHD thixotropic nanofluid past a vertical surface coexisting with both nanoparticles and gyrotactic microorganisms, Scientific Reports, vol. 11, no. 1, pp. 1–15, 2021. doi: 10.1038/s41598-020-79139-8 34404877PMC8371174

[21] PuneethV., ManjunathaS., and GireeshaB., Quartic autocatalysis of homogeneous and heterogeneous reactions in the bioconvective flow of radiating micropolar nanofluid between parallel plates, Heat Transfer, vol. 50, no. 6, pp. 5925–5950, 2021.

[22] AzamM., XuT., MaboodF., and KhanM., Non-linear radiative bioconvection flow of cross nano-material with gyrotatic microorganisms and activation energy, International Communications in Heat and Mass Transfer, vol. 127, p. 105530, 2021.

[23] Chandra Shekar BallaRamesh Alluguvelli, NaikotiKishan, Oluwole Daniel Makinde, Effect of Chemical Reaction on Bioconvective Flow in Oxytactic Microorganisms Suspended Porous Cavity, J. Appl. Comput. Mech., 6(3) (2020) 653–664

[24] MakindeO.D., AnimasaunI.L., Bioconvection in MHD nanofluid flow with nonlinear thermal radiation and quartic autocatalysis chemical reaction past an upper surface of a paraboloid of revolution, International Journal of Thermal Sciences, Volume 109, November 2016, Pages 159–171

[25] MakindeO.D., AnimasaunI.L., Thermophoresis and Brownian motion effects on MHD bioconvection of nanofluid with nonlinear thermal radiation and quartic chemical reaction past an upper horizontal surface of a paraboloid of revolution, Journal of Molecular Liquids, Volume 221, September 2016, Pages 733–743

[26] KhanW.A., MakindeO.D., KhanZ.H., MHD boundary layer flow of a nanofluid containing gyrotactic microorganisms past a vertical plate with Navier slip, International Journal of Heat and Mass Transfer, Volume 74, July 2014, Pages 285–291

[27] KhanW.A., MakindeO.D., MHD nanofluid bioconvection due to gyrotactic microorganisms over a convectively heat stretching sheet, International Journal of Thermal Sciences, Volume 81, July 2014, Pages 118–124

[28] BahiraeiM., Impact of thermophoresis on nanoparticle distribution in nanofluids, Results in Physics, vol. 7, pp. pages 136–138, 2017.

[29] SheikholeslamiM., JaliliP., and GanjiD., Magnetic field effect on nanofluid flow between two circular cylinders using agm, Alexandria Engineering Journal, vol. 57, no. 2, pp. 587–594, 2018.

[30] MirzaeyanM. and ToghraieD., Numerical investigation of laminar heat transfer and nanofluid flow between two porous horizontal concentric cylinders, Journal of Central South University, vol. 26, no. 7, pp. 1976–1999, 2019.

[31] ArifM., KumamP., KhanD., and WatthayuW., Thermal performance of go-mos2/engine oil as maxwell hybrid nanofluid flow with heat transfer in oscillating vertical cylinder, Case Studies in Thermal Engineering, vol. 27, p. 101290, 2021.

[32] AbbasN., NadeemS., SaleemA., MalikM., IssakhovA., and AlharbiF. M., Models base study of inclined mhd of hybrid nanofluid flow over nonlinear stretching cylinder, Chinese Journal of Physics, vol. 69, pp. 109–117, 2021.

[33] ReddyP. S., SreedeviP., and ChamkhaA. J., Heat and mass transfer analysis of nanofluid flow over swirling cylinder with cattaneo—christov heat flux, Journal of Thermal Analysis and Calorimetry, pp. 1–16, 2021.

[34] BiswalU., ChakravertyS., OjhaB. K., and HusseinA. K., Numerical simulation of magnetohydrodynamics nanofluid flow in a semi-porous channel with a new approach in the least square method, International Communications in Heat and Mass Transfer, vol. 121, p. 105085, 2021.

[35] KhanA., SaeedA., GulT., MukhtarS., AliI., and JawadM., Radiative swirl motion of hydromagnetic casson nanofluid flow over rotary cylinder using joule dissipation impact, Physica Scripta, vol. 96, no. 4, p. 045206, 2021.

[36] AghamiriH., NiknejadiM., and ToghraieD., Analysis of the forced convection of two-phase ferronanofluid flow in a completely porous microchannel containing rotating cylinders, Scientific Reports, vol. 11, no. 1, pp. 1–18, 2021. doi: 10.1038/s41598-020-79139-8 34497293PMC8426404

[37] BouzerzourA., TayebiT., ChamkhaA. J., and DjezzarM., Numerical investigation of natural convection nanofluid flow in an annular space between confocal elliptic cylinders at various geometrical orientations, Computational Thermal Sciences: An International Journal, vol. 12, no. 2, 2020.

[38] ChuYu-Ming, KhanNargis, M. Ijaz Khan, Kamel Al-Khaled, Nasreen Abbas, Sami Ullah Khan, et al, Thermophoresis particle deposition analysis for nonlinear thermally developed flow of Magneto-Walter’s B nanofluid with buoyancy forces, Alexandria Engineering Journal, Volume 60, Issue 1, February (2021), pp. 1851–1860.

[39] Sami Ullah Khan and Hafiz Muhammad Ali, Swimming of gyrotactic microorganisms in unsteady flow of Eyring Powell nanofluid with variable thermal features: Some bio-technology applications, International Journal of Thermophysics, 41, Article number: 159 (2020).

[40] Sami Ullah KhanKamel Al-Khaled and M. Ijaz Khan, Convective nonlinear thermally developed flow of thixotropic nanoliquid configured by Riga surface with gyrotactic microorganism and activation energy: A bio-technology and thermal extrusion model, International Communications in Heat and Mass Transfer, Volume 119, December 2020, 104966, (2020).

[41] LaidoudiHoussem, AmeurHouari, Investigation of the mixed convection of power-law fluids between two horizontal concentric cylinders: Effect of various operating conditions, Thermal Science and Engineering Progress, Volume 20, 1 December 2020, 100731

[42] MokeddemMourad, LaidoudiHoussem, Oluwole Daniel MakindeMohamed Bouzit, 3D Simulation of Incompressible Poiseuille Flow through 180° Curved Duct of Square Cross-section under Effect of Thermal Buoyancy, Periodica Polytechnica Mechanical Engineering, 63(4), pp. 257–269, 2019.

[43] LaidoudiH. (2020). Enhancement of natural convection heat transfer in concentric annular space using inclined elliptical cylinder. Journal of Naval Architecture and Marine Engineering, 17(2), 89–99.

[44] LaidoudiHoussem, OluwoleDaniel Makinde, Mixed Convection Heat Transfer around a Tandem Circular Cylinders in Incompressible Downward Flow, Diffusion Foundations (Volume 16), 12–20

[45] HoussemL., MustaphaH., MohamedB. and AbdellahG., Natural-convection of Newtonian fluids between two concentric cylinders of a special cross-sectional form, Thermal Science 2021 Volume 25, Issue 5 Part B, Pages: 3701–3714.

[46] HosnyAbou-Ziyan1, Reda Ameen1 and Khairy Elsayed, Fluid flow and convection heat transfer in concentric and eccentric cylindrical annuli of different radii ratios for Taylor-Couette-Poiseuille flow, Advances in Mechanical Engineering 2021, Vol. 13(8) 1–22.

[47] NazeerM., HussainF., KhanM. I., RehmanA. U., El-ZaharE. R., ChuY. M., et al, Theoretical study of MHD electro-osmotically flow of third-grade fluid in micro channel, Appl. Math. Comput., 420 (2022) 126868.

[48] ChuY. M., ShankaralingappaB. M., GireeshaB. J., AlzahraniF., KhanM. I. and KhanS. U., Combined impact of Cattaneo-Christov double diffusion and radiative heat flux on bio-convective flow of Maxwell liquid configured by a stretched nano-material surface, Appl. Math. Comput., 419 (2022) 126883.

[49] ZhaoT.-H., KhanM. I. and ChuY.-M., Artificial neural networking (ANN) analysis for heat and entropy generation in flow of non-Newtonian fluid between two rotating disks, Math. Methods Appl. Sci., 2021. 10.1002/mma.7310.

[50] IqbalM. A., WangY., MiahM. M., OsmanM. S., Study on Date–Jimbo–Kashiwara–Miwa Equation with Conformable Derivative Dependent on Time Parameter to Find the Exact Dynamic Wave Solutions, Fractal Fract., 2022, 6(1), Article 4, 12 pages. 10.3390/fractalfract6010004

